# Selection of the Male or Female Sex in Chronic Unpredictable Mild Stress-Induced Animal Models of Depression

This article has been retracted.

**DOI:** 10.1155/2022/2602276

**Published:** 2022-06-30

**Authors:** Shuo Jiang, Ling Lin, Lihua Guan, Youming Wu

**Affiliations:** ^1^Department of Acupuncture and Moxibustion, The First Affiliated Hospital of Zhejiang Chinese Medical University, Hangzhou, China; ^2^Department of Acupuncture and Moxibustion, Quzhou Hospital of Traditional Chinese Medicine, Quzhou, China; ^3^Department of Acupuncture and Moxibustion, Quzhou TCM Hospital at the Junction of Four Provinces Affiliated to Zhejiang Chinese Medical University, Quzhou, China

## Abstract

Depression is a serious public health problem and an important factor leading to disease-related disability. Influenced by many factors, such as psychological, hormonal, and genetic factors, the incidence rate of depression in females is approximately two times that in males. However, in preclinical neuroscience research, the selection of the animals' sex for use in depression models has been controversial. At present, in most preclinical studies, the animals generally chosen in depression models have been male rodents rather than female rodents. It remains doubtful whether the data obtained from male animals can be generalized to female animals. The performance of female animals in preclinical studies of depression has been inconclusive. Based on a review of a large number of original studies in the PubMed database, it was found that although male rodents are more commonly used in the study of depression, the use of female animals also shows good modeling of depression and has its advantages. The influence of the animals' sex in the chronic unpredictable mild stress (CUMS) model needs further research.

## 1. Introduction

Depression is a common psychoaffective disorder characterized by a depressed mood, loss of interest, reduced speech activity, inability to enjoy life, and even suicidal thoughts. According to data from the World Health Organization, nearly 300 million people worldwide suffer from depression [1]. The number of sudden cases of depression in the world increased by 49.86% in 2017 compared with that in 1990 [2]. Depression is an important public health problem and the biggest factor leading to disease-related disability. Globally, depression accounts for 5.6% of disability-adjusted life years in women and 4.3% in men [3]. The rate of depression in women is approximately twice that in men [4].

Women's susceptibility to depression is considered to be related to a variety of factors, such as psychological, neurochemical, anatomical, hormonal, genetic, and personality factors [5]. There are sex differences in women's susceptibility to stress, anxiety, and depression. Studies have found that many aspects of brain function show important gender differences, which affect behavior, mental health, and mental disorders. Autopsies of male and female patients diagnosed with major depression disorder showed significant gender differences in multiple brain regions [6]. The occurrence of depression is related to an increase in hippocampal neuritis [7]. The low anti-inflammatory capacity and strong stress response in the female hippocampus may lead to gender differences in depression. The nucleus accumbens is an area of the brain that integrates pleasure experience and emotional processing. There is a significant overlap in gender-specific regulation of immune-related genes in the nucleus accumbens in male and female mice [8, 9].

There are differences between female and male rodents in depression models. Male and female Sprague–Dawley rats exposed to chronic mild stress had different sensitivities to chronic mild stress, and female rats were more vulnerable to HPA axis imbalance with exposure to chronic mild stress [10]. When male and female rats were exposed to the same stressor, female rats seemed to be more vulnerable to neuroendocrine and behavioral changes [11]. When male and female mice were subjected to chronic unpredictable mild stress (CUMS) for 4 weeks, behavioral tests used to assess depression-like behavior found that weight gain, sucrose preference, and spontaneous activity were disrupted in both sexes. However, these effects were often larger in females [12]. Female rodents are more sensitive to chronic stress and may be more appropriate for the study of depression.

In rodents, the CUMS procedure has been used to simulate conditions leading to the behavioral and physiological consequences of chronic stress [13]. Animals exposed to chronic stress often exhibit significant depressive behavioral deficits, such as loss of pleasure, helplessness, cognitive impairment, and anxiety [14, 15]. Although a few studies have shown gender differences between animal model systems and humans, most preclinical translational neuroscience experiments use only male mice or rats [16–18]. Generally, male animals have attracted attention for use in animal models because of concerns about the confounding factors of hormone cycle changes in female animals. However, studies have shown that in most situations, the variability observed in female mice across the whole hormone cycle is not greater than that of male mice [19]. Moreover, the data obtained in male animals may not be generalizable to the psychopathology and efficacy of drug therapy in female animals [20].

In 2014, the United States National Institutes of Health noted the impact of gender differences on research and puts forward a series of suggestions [21]. In particular, it was suggested that more attention should be given to gender differences in the study of depression as there is a high incidence rate in women. Taking the animal model of depression caused by CUMS as an example, this paper evaluated the use of female or male animals in preclinical research, analyzed its causes, and provided some guidance and suggestions.

## 2. Methods

### 2.1. Search Strategies

We searched the PubMed database. The following search phrase was used: “((((rat [Title/Abstract]) OR (mice [Title/Abstract])) AND (depression [MeSH Terms])) AND (CUMS[Title/Abstract])) AND ((“2002/01/01 “[Date - Publication]:” 2021/12/31 “[Date - Publication])).”

### 2.2. Eligibility Criteria

The analysis included studies that met the following criteria: (1) animal studies of models that established depressive-like behaviors; (2) the model animals being female rats or mice, without diabetes, hypertension, transgenes, and other basic diseases; (3) the depression model being established by the CUMS procedure; and (4) outcome indicators including evaluation of depressive-like behavior. Included studies do not include human studies, case reports, cell studies, and reviews. Female-related depression, such as postpartum depressive disorders and perimenopausal depression, which must use female animals was excluded.

### 2.3. Data Extraction

The following details were extracted from the relevant research by two independent authors: (1) the name of the first author and the year of publication of the paper; (2) animal information, including species, sex, weight, and age; (3) the time for CUMS to establish depressive-like behavior model; and (4) related indicators for evaluating depressive-like behavior.

### 2.4. Methodological Quality of Studies

The methodological quality of the included studies was assessed using the 10-item scale with minor modification [22, 23]. The contents of the 10-item scale were as follows: (a) peer-reviewed publications, (b) control temperature, (c) randomization of the experiment, (d) blind methods for model induction, (e) blinded outcome assessments, (f) anesthetics without significant intrinsic cardioprotective effects, (g) appropriate animal models (elderly, diabetic, or hypertensive animals), (h) sample size calculation, (i) compliance with animal welfare regulations, and (j) potential conflict of interest statements. In the included studies, 1 item mentioned was counted as 1 point. A maximum of 10 points might be obtained for each study. Two independent researchers completed the scoring of the included study.

### 2.5. Statistical Analysis

Endnote x9 was used to save the articles finally included in the study and establish a database. Microsoft Office Excel 2016 was used to create tables and record the extracted data, including the author, title, year of publication, animal species, weight, age, CUMS exposure time, and evaluation index.

## 3. Results

### 3.1. Study Selection

A total of 457 articles were found by searching the PubMed database. Based on an Endnote X9.0 quick search of “female,” 417 articles were excluded. We analyzed the remaining 40 articles and then deleted 17 articles for the following reasons: (1) full text was not available; (2) CUMS model animals were male; (3) there was an unclear research plan; and (4) the article was an overview. The remaining 23 articles were read in full, and the articles studying diseases that must be examined with female rats were excluded. These diseases included (1) postpartum depressive disorders [24, 25] and (2) perimenopausal depression [26–30], and 16 studies were ultimately selected [12, 31–45] (Figure 1).

### 3.2. Study Quality

The detailed results of the quality of the included studies are shown in Table 1. The maximal total score of the study quality is 10, and the study quality included in the study ranges from 3 to 6. Two studies scored 3 [39, 40]; 6 studies scored either 4 [31, 32, 36, 42–44] or 5 [33, 35, 37, 38, 41, 45]; and 2 studies scored 6 [12, 34]. All the included studies were in compliance with animal welfare regulations. All the studies were conducted on healthy rats or mice and randomly divided into groups, but there was no sample size calculation. All studies did not have blind modeling, and only two studies had blind evaluation. All publications are peer reviewed. The temperature was controlled in 14 studies. Fifteen studies stated that there were no potential conflicts of interest.

### 3.3. Characteristics of the Included Studies

A total of 16 papers were included in this study. The authors of 11 papers were from China [12, 31, 33–36, 38, 41, 43–45], the authors of 2 papers were from India [39, 40], and the authors of one paper were from the United States [42], as well as one from Brazil [32] and one from Egypt [37]. One study was published in 2021 [41], three in 2020 [31, 35, 38], six in 2019 [12, 37, 42–45], and three in 2018 [33, 34, 40]. There was one study published in 2013, one in 2015, and one in 2017. In all studies, female animals were exposed to the CUMS procedure to establish depression models. All studies had corresponding evaluation indices of depressive behavior after the CUMS procedure. Animals were exposed to a variety of stressors during the CUMS procedure. The same source of stress could not be used continuously. Animals were exposed to the CUMS procedure for 28 days in 6 studies [12, 31, 33, 34, 39, 40]. Animals in two studies were exposed to the CUMS procedure for 21 days [36, 37], in two studies for 42 days [43, 45], and in two studies for 45 days [38, 44]. There was one study that exposed animals to the CUMS procedure for 14 days, for 35 days, for 56 days, and for 70 days [33, 35, 41, 42]. The general characteristics of the listed publications are shown in Tables 2 and 3.

### 3.4. Animals Exposed to the CUMS Procedure

Among the 16 studies, 8 studies used rats to establish a CUMS depression model and 9 studies used mice to establish a CUMS depression model. Among them, the CUMS depression model in one study used female Kunming mice and female Sprague–Dawley rats at the same time [34]. The rats in these studies were all female Sprague–Dawley rats. Three studies used both female and male rats [36, 41, 42], and one study used both female and male mice [12]. The weight of the rats ranged from 170 to 300 g, and the age ranged from 8 weeks to 12 weeks. There were three studies with the CUMS depression model that used female C57BL/6J mice [31, 33, 45], two used female C57BL/6 mice [12, 35], two used female Swiss Albino mice [39, 40], one used female BALB/c mice [37], and one used female Kunming mice [34]. The weight of the mice ranged from 12 to 30 g, and their ages ranged from 49 to 90 days.

### 3.5. Indicators for Evaluating the Depression Model

After the animals were exposed to the CUMS procedure to establish a model of depression, all studies evaluated depressive behavior. The sucrose preference test was the most widely used procedure, and most studies adopted it. Eleven studies [12, 31–33, 35, 36, 38, 40–43] used the open field test to evaluate the depressive behavior of CUMS model animals, and 10 studies [31, 32, 34, 35, 37–40, 44, 45] used the forced swimming test. Four studies [12, 31, 34, 45] conducted the tail suspension test in the CUMS model, three studies [34, 36, 42] observed changes in body weight, two studies [34, 37] assessed the locomotor activity, and two studies [35, 44] measured the performance in the elevated plus maze test. The light and dark box test, self-grooming behaviors, social interaction test, despair-like behavior in fear conditioning chamber, and splash test were each tested in only one study in the evaluation of the depressive behavior of animals after exposure to the CUMS procedure.

## 4. Discussion

This research showed that some studies using the CUMS model of depression chose female animals, although most studies use male animals to establish the CUMS depression model. A total of 9 studies used female mice to establish a CUMS depression model, and 8 studies used female rats to establish a CUMS depression model; one of these studies used both female rats and female mice. Although depression is more common in women than men, more males than females have been used in animal studies.

Researchers have developed several animal models to simulate depression, such as CUMS, chronic immobilization stress, chronic social failure stress, early life stress, and chronic restraint stress, each of which has been used to induce depression-like behavior [46–48]. Among them, CUMS is widely used to induce depression-like behavior in rodents to study the biological mechanisms underlying depression. In the CUMS procedure, animals are exposed to different types of mild stress every day, which simulates chronic stressful life events, resulting in decreased pleasure and energy. The CUMS depression model is the most commonly used, reliable, and effective rodent depression model [49].

At present, male rodents are widely used in chronic unpredictable stress models [50]. Sex is a determinant of susceptibility to CUMS-induced depressive behavior, and male rodents are more vulnerable to chronic stress-induced neuronal damage and behavioral defects [12, 51]. Chronic stress can lead to profound changes in the morphology of neurons in the medial prefrontal cortex of male rats. In male rats, stress reduces the number and length of dendritic apical branches, while in female rats, stress increases the length of dendritic apical branches [52]. When female and male Sprague–Dawley rats were exposed to the CUMS procedure, it was evident from depressive behavior and monoamine neurotransmitter levels that it was more difficult for male rats to tolerate stress than female rats [41]. After chronic stress, men show memory impairments, while women show cognitive resilience to chronic stressors; consequently, men's cognitive function assessed through spatial tasks is damaged, and women's memory is not affected by stress [53]. The CUMS procedure only induced depression-like behavior in male rats on day 28. In males, the CUMS procedure on day 28 reduced sucrose consumption in the sucrose preference test, increased immobility time in the forced swimming test, and increased the time that rats spent in the center of the activity field, indicating that the change in motor activity induced by exposure to CUMS occurred in a sex-dependent manner and that male rats were more vulnerable to CUMS than female rats [54].

Some conflicting reports have shown that female mice are more sensitive to the CUMS procedure and the CUMS procedure has different effects on the behavior of male and female mice. Compared with male mice, female mice experience slower weight gain and faster weight loss when exposed to the CUMS procedure. The decrease in sucrose preference and central activity duration in female mice was greater than that in male mice. Exposure to the CUMS procedure increased the depression-related behavior and decreased serum BDNF in female rats but not in male rats [42]. After stress, the changes in TNF-*α*/IL-10 and iNOS/Arg-1 in female mice were more obvious. The expression of BDNF and its receptor TrkB in the hippocampus of female mice was significantly decreased compared with that in the hippocampus of male mice [12]. Some studies have shown that some depressive behaviors occur only in female animals. Early-life stress induced depression-like behavior in female mice but not in male mice [48]. Research has shown that BDNF/TrkB, especially GSK3/*β*-catenin, activates signaling pathways such that the role of D1-D2 heteromers in promoting antidepressant and anxiety-promoting effects is more obvious in female rats than in male rats [55]. After the CUMS procedure, female rats showed more severe depression-like behavior than male rats [56]. Compared with female rats, male rats showed more biological changes related to anxiety and depression.

The application of the CUMS depression model in female animals achieved good modeling effects. Female wild-type C57BL/6J mice exposed to the CUMS procedure exhibited increased depression-like behavior, which was manifested by increased immobility time in the forced swimming and tail suspension tests, reduced sucrose preference in the sucrose preference test, and reduced the exploratory behavior in the open field test [31]. Exposure of female wild-type C57BL/6J mice to the CUMS procedure induced/increased sucrose preference, field exploration, social interaction, entries into and time spent in the open arms of the elevated plus maze, and immobility time in the forced swimming test [35]. Behavioral tests, such as the sucrose preference test, forced swimming test, and fear conditioned reflex, have been used to evaluate depression-like behavior in mice. It was found that female mice exposed to CUMS exhibited reduced sucrose consumption, prolonged resting time in the forced swimming test, and increased defensive freezing time in the fear conditioned reflex test, which are clear expressions of depression-like behavior [37]. Exposure of female mice to the CUMS procedure for 28 days significantly reduced sucrose preference, combing behavior in the splash test, body weight, and immobility in the forced swimming test [39]. The abovementioned studies show that clear depressive behaviors can be induced in female rats or mice with the CUMS procedure.

Female wild-type C57BL/6J mice exposed to the CUMS procedure showed significant decreases in the levels of BDNF and NGF and the activities of Na^+^ and K^+^-ATPase, decreased levels of the nonprotein mercaptan, and increased levels of reactive oxygen species. Glutathione reductase, glutathione peroxidase, and catalase activities increased in mice exposed to the CUMS procedure [32]. After female mice were exposed to the CUMS procedure, the levels of BDNF, 5-HT, NE, and DA decreased, the levels of serum corticosterone, IL-6, and TNF-*α* increased, and there was an imbalance in oxidative antioxidants in the hippocampus and cerebral cortex [40]. After adult female Sprague–Dawley rats were exposed to the CUMS procedure for six weeks, the expression of the microglial M1 markers CD11b, TNF-*α*, INF-*γ*, IL-1*β*, and IL-17 increased but the M2 cytokine concentrations of IL-4, IL-10, and IL-13 decreased. At the same time, CUMS inhibited the expression of astrocyte markers glial fibrillary acidic protein, brain-derived neurotrophic factor, and TrkB [44]. After female rats were exposed to the CUMS procedure, the expression of the proinflammatory cytokines IL-1*β*, IL-6, and TNF-*α* in the hippocampus increased and the expression of BDNF, GDNF, and NGF decreased. CUMS exposure also stimulated the HPA axis to release more corticosterone and led to 5-HT and NE defects in the hippocampus [38]. The abovementioned studies show that female rats or mice have obvious changes in biological indicators in the CUMS-induced depression model, which can be useful in the preclinical study of depression.

## 5. Conclusion

Male rodents are more commonly used in the CUMS model of depression, but female rats or mice also show stable changes in depression-like behavior and biological indicators. Female rats or mice can be used in the CUMS model of depression, although there are still some inconsistencies, and further research is needed.

## Figures and Tables

**Figure 1:** Summary of the process for identifying candidate studies.

**Table 1:** Methodological quality for each included study.

Study	a	b	c	d	e	f	g	h	i	j	Total
Cheng et al. [31]	+	+	—	—	—	—	—	—	+	+	4
Filho et al. [32]	+	+	—	—	—	—	—	—	+	+	4
Fu et al. [33]	+	+	+	—	—	—	—	—	+	+	5
He et al. [34]	+	+	+	—	+	—	—	—	+	+	6
Li et al. [35]	+	+	+	—	—	—	—	—	+	+	5
Liu et al. [12]	+	+	+	—	—	+	—	—	+	+	6
Lu et al. [36]	+	—	+	—	—	—	—	—	+	+	4
Mahmoud et al. [37]	+	+	+	—	—	—	—	—	+	+	5
Peng et al. [38]	+	+	—	—	+	—	—	—	+	+	5
Taksande et al. 2013 [39]	+	+	—	—	—	—	—	—	+	—	3
Thakare et al. [40]	+	—	—	—	—	—	—	—	+	+	3
Wang et al. [41]	+	+	+	—	—	—	—	—	+	+	5
Weisbrod et al. [42]	+	+	—	—	—	—	—	—	+	+	4
Zhang et al. [43]	+	+	—	—	—	—	—	—	+	+	4
Zhang et al. [44]	+	+	—	—	—	—	—	—	+	+	4
Zhou et al. [45]	+	+	+	—	—	—	—	—	+	+	5

**Table 2:** Depression model induced by the CUMS procedure in female mice.

Study	Animal	Body weight/age	CUMS exposure time	Depression evaluation
Cheng et al., 2020	C57BL/6J mice	12–20 g, 7–9 weeks	28 days	Forced swimming test, tail suspension test, sucrose preference test, open field test
Filho et al., 2015	C57BL/6J mice	20–25 g, 90 days	28 days	Sucrose preference test, forced swimming test, open field test
He et al., 2018	Kunming mice	20–25 g	28 days	Forced swimming test, tail suspension test, locomotor activity
Li et al., 2020	C57BL/6 mice	21 ± 2 g; 8 weeks	56 days	Sucrose preference test, elevated plus maze, open field test, forced swimming test, social interaction test
Liu et al., 2019	C57BL/6 mice	18–22 g, 8 weeks	28 days	Sucrose preference test, tail suspension test, open field test
Mahmoud et al., 2019	BALB/c mice	22 ± 2.5 g, 7 weeks	21 days	Sucrose preference test, forced swim test (FST), despair-like behavior in fear conditioning chamber, locomotor activity
Taksande et al., 2013	Swiss albino mice	25–30 g, adult	28 days	Sucrose preference test, splash test, forced swim test
Thakare et al., 2018	Swiss albino mice	30–35 g, 70–80 days	28 days	Sucrose preference test, forced swim test, open field test
Zhou et al., 2019	C57BL/6J mice	18–22 g, 8 weeks	42 days	Sucrose preference test, forced swimming test, and tail suspension test

**Table 3:** Depression model induced by the CUMS procedure in female rats.

Study	Animal	Body weight/age	CUMS exposure time	Depression evaluation
Fu et al., 2018	Sprague–Dawley rats	238 ± 26 g, 12 weeks	35 days	Open field test, sucrose consumption test.
He et al., 2018	Sprague–Dawley rats	170–180 g	28 days	Body weight, sucrose intake changes
Lu et al., 2017	Sprague–Dawley rats	230–250 g, 8 weeks	21 days	Body weight, open field test, sucrose preference test
Peng et al., 2020	Sprague–Dawley rats	280–300 g, 8–12 weeks	45 days	Sucrose preference test, forced swimming test, open field test
Wang et al., 2021	Sprague–Dawley rats	200–220 g	70 days	Sucrose preference test, light and dark box test (LDB), open field test
Weisbrod et al., 2019	Sprague–Dawley rats	51–55 d	14 days	Open field activity, body weight
Zhang et al., 2019	Sprague–Dawley rats	250–280 g, adult	42 days	Open field test, self-grooming behaviors
Zhang et al., 2019	Sprague–Dawley rats	250–280 g, adult	45 days	Sucrose preference test, forced swimming test, elevated plus maze test

## Data Availability

The raw data used to support the findings of this study are available from the corresponding author upon request.
